The article "Differential Human Learning Optimization Algorithm" was published in 2022. Journal: Comput Intell Neurosci.

# Differential Human Learning Optimization Algorithm

**DOI:** 10.1155/2022/5699472

**Published:** 2022-04-30

**Authors:** Pinggai Zhang, Ling Wang, Jiaojie Du, Zixiang Fei, Song Ye, Minrui Fei, Panos M. Pardalos

**Affiliations:** ^1^Industrial Process Control Optimization and Automation Engineering Research Center, School of Electronic Engineering, Chaohu University, Chaohu, Anhui 238024, China; ^2^Shanghai Key Laboratory of Power Station Automation Technology, School of Mechatronics Engineering and Automation, Shanghai University, Shanghai 200444, China; ^3^School of Computer Engineering and Science, Shanghai University, Shanghai 200444, China; ^4^Center for Applied Optimization, Department of Industrial and Systems Engineering, University of Florida, Gainesville, FL 32611, USA

## Abstract

Human Learning Optimization (HLO) is an efficient metaheuristic algorithm in which three learning operators, i.e., the random learning operator, the individual learning operator, and the social learning operator, are developed to search for optima by mimicking the learning behaviors of humans. In fact, people not only learn from global optimization but also learn from the best solution of other individuals in the real life, and the operators of Differential Evolution are updated based on the optima of other individuals. Inspired by these facts, this paper proposes two novel differential human learning optimization algorithms (DEHLOs), into which the Differential Evolution strategy is introduced to enhance the optimization ability of the algorithm. And the two optimization algorithms, based on improving the HLO from individual and population, are named DEHLO1 and DEHLO2, respectively. The multidimensional knapsack problems are adopted as benchmark problems to validate the performance of DEHLOs, and the results are compared with the standard HLO and Modified Binary Differential Evolution (MBDE) as well as other state-of-the-art metaheuristics. The experimental results demonstrate that the developed DEHLOs significantly outperform other algorithms and the DEHLO2 achieves the best overall performance on various problems.

## 1. Introduction

In the past decades, traditional optimization algorithms are widely used in science, engineering, economics, and industry to solve optimization problems [1]. However, the traditional optimization algorithms need to learn the mathematical characteristics of the optimal solution in advance, which can result in added complexity in the algorithm's designation. In addition, the traditional algorithms cannot escape the local optimal of complex problems effectively. With the development of technology, engineering problems with optimization objectives are becoming more and more complicated and the conventional algorithm to solve the NP problems has become very difficult, which forces researchers to study metaheuristic algorithms [2]. Metaheuristics are general frameworks to build heuristics for combinatorial and global optimization problems [3]. The application of natural or biology-inspired metaheuristic optimizations, such as Genetic Algorithm [4], Particle Swarm Optimization [5], Harmony Search [6], Differential Evolution (DE) [7–10], Artificial Bee Colony [11], Fruit Fly Optimization [12], Distributed Grey Wolf Optimizer (DGWO) [13], Moth Search Algorithm (MSA) [14], Slime Mould Algorithm (SMA) [15], Gaining Sharing Knowledge-Based Optimization [16, 17], Cuckoo Search with Exploratory (ECS) [18], Discrete Jaya with Refraction Learning and Three Mutation (DJRL3M) [19], and Monarch Butterfly Optimization (MBO) [20], Hunger Games Search (HGS) [21], Runge Kutta Method (RUN) [22], and Harris Hawks Optimization (HHO) [23], has been very successful to solve the complex optimization problems, such as feature selection [24–28], image segmentation [29], controller designation [30], flow-shop scheduling problem [31, 32], and the node placement of wireless sensor networks [33].

The article "Differential Human Learning Optimization Algorithm" was published in 2022. Journal: Comput Intell Neurosci.

Human beings are the smartest creature in the world because of their strongest learning ability; they are smarter than other living beings, such as birds, ants, and fish. To solve complex problems effectively, humans are always repetitively learning to improve their skills for adapting to the external environment better. Many human learning activities are similar to the search process of metaheuristics. For example, when a person learns something new, he or she repeatedly practices to improve new skills and evaluates his or her performance for guiding the following study. The process of human learning just like the metaheuristic algorithms iteratively generates a new solution and calculates the corresponding fitness for adjusting the following search. Therefore, it is reasonable to consider that the metaheuristic algorithm based on the human learning mechanisms may have advantages over other biological systems-based algorithms on complicated problems. Inspired by this thought, Wang et al. [34] proposed the Human Learning Optimization Algorithm (HLO) based on a simplified human learning model, in which three learning operators, i.e., the random learning operator (RLO), the individual learning operator (ILO), and the social learning operator (SLO), are developed to search out the optimal solution, which represents that a person may learn randomly due to the lack of prior knowledge or exploring new strategies, learn from his or her previous experience, and learn from his or her friends and books, respectively.

The article "Differential Human Learning Optimization Algorithm" was published in 2022. Journal: Comput Intell Neurosci.

To strengthen the search efficiency of HLO, a few enhanced variants have been subsequently developed. An adaptive simplified human learning optimization algorithm (ASHLO) [35] is proposed in which the pr and pi, two control parameters determining the rates of performing RLO, ILO, and SLO, are linearly adjusted to achieve the balance between the global search and local search. Encouraged by the success of ASHLO, a sine-cosine adaptive human learning optimization algorithm (SCHLO) [36] is proposed in which the pr and pi are dynamically tuned in a reasonable range by the sine and cosine functions so that SCHLO can efficiently escape from the local optimal. Later, a new improved adaptive human learning optimization algorithm (IAHLO) [37] is presented to accurately tune the control parameter pr so that IAHLO can keep the diversity better at the early stage and perform the local search more efficiently at the later stages of iterations. Besides, inspired by the intelligence quotient (IQ) of humans, a diverse human learning optimization algorithm (DHLO) [38] is presented in which the control parameter pi is initialized by a Gaussian distribution and dynamically adjusted according to the pi value of the best individual. To further extend HLO, a novel hybrid-coded HLO (HcHLO) [39] is proposed to tackle mix-coded problems, in which real-coded parameters are optimized by a new continuous HLO (CHLO) [39] and the binary and discrete variables are handled by the binary learning operators of HLO. Until now, HLO has been successfully applied to engineering design problems [37], knapsack problems [40], optimal power flow calculation [41], extractive text summarization [42], financial markets forecasting [43], furnace flame recognition [44], scheduling problems [45], and intelligent control [46]. In particular, HLO obtained the best-so-far results on two well-studied sets of multidimensional knapsack problems, i.e., 5.100 and 10.100 [40], as well as the set of mixed-variable optimization problems [39] which implies the promising advantages of HLO.

In HLO, social learning adopts the greedy strategy to generate a new candidate, i.e., simply yet efficient copying the bit value from the SKD, which makes the algorithm easy to fall into local optimal. So, the relearning operator is introduced into HLO [40] to help the algorithm to escape from the local optimal. However, the relearning operator may destroy the existing optimal information, which further reduces the performance of the algorithm. On the other hand, the social learning of the HLO just learns from the global solution, which is inconsistent with the actual society. In real life, people could learn from the best solution of other individuals in the population. The Modified Binary Differential Evolution (MBDE, modified binary DE which is the previous work) [47] reverses the updating strategy of the standard Differential Evolution (DE) [7] so that DE can better keep the robustness of parameter settings and the diversity of the population to search for optimal bit information effectively. Therefore, this paper proposes two novel differential human learning optimization algorithms (DEHLOs), in which the strategy of MBDE is introduced into HLO to further improve the performance of DEHLOs algorithm by using the optimal information of other individuals.

The article "Differential Human Learning Optimization Algorithm" was published in 2022. Journal: Comput Intell Neurosci.

This paper is organized as follows.  Section 2 gives a brief review of the HLO and MBDE, respectively.  Section 3 presents the concepts, operators, and implementation of the proposed DEHLO1 and DEHLO2 in detail.  Section 4 verified that the proposed DEHLOs have significant advantages over the compared algorithms on the multidimensional knapsack problems. Finally, conclusions are drawn in Section 5.

## 2. Related Works

### 2.1. Human Learning Optimization

The HLO adopts the binary-coding framework, and consequently an individual in HLO is represented by a binary string as

(1) $$\begin{array}{c} x_{i}=\left[\begin{array}{cccccc} x_{i1} & x_{i2} & \ldots & x_{ij} & \ldots & x_{iM} \end{array}\right],\\ x_{ij}\in \left\{0,1\right\},\\ 1\leq i\leq N,\\ 1\leq j\leq M, \end{array}$$

where *x*_*i*_ denotes the *i*-th individual, *N* is the size of the population, and *M* is the dimension of solutions. Each bit of binary string is initialized as “0” or “1” randomly.

Random learning operator: At the beginning of the learning process, people always keep exploring new strategies to solve problems because there is no prior knowledge [48]. Besides, an individual cannot fully replicate their previous experience and social knowledge because of the disturbance of external and forgetting. To emulate these phenomena of human random learning, the HLO executes random learning operator (RLO) with a certain probability as

(2) $$\begin{array}{c} x_{ij}=RE\left(0,1\right)=\left\{\begin{array}{cc} 0, & r_{1}\leq 0.5,\\ 1, & \text{else,} \end{array}\right. \end{array}$$

where *r*_1_ is a stochastic number between 0 and 1.

Individual learning operator: Individual learning is defined as the ability to build knowledge through individual reflection about external stimuli and sources [49], which could be regarded as individual behavior in the trial and error process of continuous improvement. To mimic human individual learning, the best individual solutions are reserved in the individual knowledge database (IKD) as

(3) $$\begin{array}{c} {\text{IKD}}_{i}=\left[\begin{array}{c} \begin{array}{c} ikd_{i1}\\ ikd_{i2} \end{array}\\ \begin{array}{c} \vdots \\ ikd_{ip} \end{array}\\ \begin{array}{c} \vdots \\ ikd_{iK} \end{array} \end{array}\right]=\left[\begin{array}{cccc} ik_{i1,1} & ik_{i1,2} & \cdots & \begin{array}{ccc} ik_{i1,j} & \cdots & ik_{i1,M} \end{array}\\ ik_{i2,1} & ik_{i2,2} & \cdots & \begin{array}{ccc} ik_{i2,j} & \cdots & ik_{i2,M} \end{array}\\ \vdots & \vdots & \vdots & \begin{array}{cccc} \vdots & \vdots & \vdots & \vdots \end{array}\\ \begin{array}{c} ik_{ip,1}\\ \vdots \\ ik_{iK,1} \end{array} & \begin{array}{c} ik_{ip,2}\\ \vdots \\ ik_{iK,2} \end{array} & \begin{array}{c} \cdots \\ \vdots \\ \cdots \end{array} & \begin{array}{ccc} \begin{array}{c} ik_{ip,j}\\ \vdots \\ ik_{iK,j} \end{array} & \begin{array}{c} \cdots \\ \vdots \\ \cdots \end{array} & \begin{array}{c} ik_{ip,M}\\ \vdots \\ ik_{iK,M} \end{array} \end{array} \end{array}\right]\text{,}\\ 1\leq i\leq N,\\ 1\leq p\leq K,\\ 1\leq j\leq M, \end{array}$$

where IKD_*i*_ denotes the individual knowledge database of the person *i*, *K* is the predefined number of solutions saved in the IKD, and *ikd*_*ip*_ represents the *p*-th best experiment of the person *i*. When HLO conducts the individual learning operator, (4) is operated to generate a new candidate solution.

(4) $$\begin{array}{c} x_{ij}=ik_{ip,j}. \end{array}$$

Social learning operator: During social learning, people can acquire knowledge and experience from other individuals to further develop their ability directly or indirectly [50], and the efficiency and effectiveness of learning will be improved from experience share [51]. To simulate the social learning of humans in HLO, the social knowledge database (SKD) is adopted to reserve the best knowledge of the population as

(5) $$\begin{array}{c} SK\;D=\left[\begin{array}{c} \begin{array}{c} skd_{1}\\ skd_{2} \end{array}\\ \begin{array}{c} \vdots \\ skd_{q} \end{array}\\ \begin{array}{c} \vdots \\ skd_{S} \end{array} \end{array}\right]=\left[\begin{array}{cccc} sk_{11} & sk_{12} & \cdots & \begin{array}{ccc} sk_{1j} & \cdots & sk_{1M} \end{array}\\ sk_{21} & sk_{22} & \cdots & \begin{array}{ccc} sk_{2j} & \cdots & sk_{2M} \end{array}\\ \vdots & \vdots & \vdots & \begin{array}{cccc} \vdots & \vdots & \vdots & \vdots \end{array}\\ \begin{array}{c} sk_{q1}\\ \vdots \\ sk_{S1} \end{array} & \begin{array}{c} sk_{q2}\\ \vdots \\ sk_{S2} \end{array} & \begin{array}{c} \cdots \\ \vdots \\ \cdots \end{array} & \begin{array}{ccc} \begin{array}{c} sk_{qj}\\ \vdots \\ sk_{Sj} \end{array} & \begin{array}{c} \cdots \\ \vdots \\ \cdots \end{array} & \begin{array}{c} sk_{qM}\\ \vdots \\ sk_{SM} \end{array} \end{array} \end{array}\right]\text{,}\\ 1\leq q\leq S,\\ 1\leq j\leq M, \end{array}$$

where *S* is the size of the SKD and *skd*_*q*_ is the *q*-th solution in the SKD. *q* is a stochastic number; it decides which one of the SKD will be used. HLO performs social learning operator as (6) to generate the new candidate solution during the search process.

(6) $$\begin{array}{c} x_{ij}=sk_{qj}. \end{array}$$

In summary, the above operators can be integrated and operated as

(7) $$\begin{array}{c} x_{ij}=\left\{\begin{array}{cc} RE\left(0,1\right), & 0\leq r\leq pr\\ ik_{ip,j}, & pr<r\leq pi\\ sk_{qj}, & \text{else,} \end{array}\right., \end{array}$$

where *r* is a stochastic number between 0 and 1, and pr and pi are the control parameters to determine the rates of HLO performing the three learning operators. Specifically, pr, (pi-pr), and (1-pi) are the probabilities of random learning, individual learning, and social learning, respectively. Algorithm 1 describes the implementation of HLO, and more details can be found in [35].

The article "Differential Human Learning Optimization Algorithm" was published in 2022. Journal: Comput Intell Neurosci.

### 2.2. Modified Binary Differential Evolution

The MBDE [47] adopts the binary-coding scheme and reserves the updating formulas of the standard DE, including the mutation operator, the crossover operator, and the selection operator. A probability estimation operator is introduced into MBDE to integrate the mutant operator.

Probability estimation operator: The probability estimation operator is used to build the probability distribution vector *f*(*p*_*i*_^*G*^) of the parent individuals. The new mutant binary individual *u*′_*ij*_^*G*^ is generated from parents' sampling randomly through the probability estimation vector as equations (8) and (9),

(8) $$\begin{array}{c} f\left(p_{ij}^{G}\right)=\frac{1}{1+e^{-\left(2b/1+2F\right)\times \left(p_{r1,j}^{G}+F\times \left(p_{r2,j}^{G}-p_{r3,j}^{G}\right)-0.5\right)}}, \end{array}$$

(9) $$\begin{array}{c} u_{ij}^{\prime G}=\left\{\begin{array}{cc} 1, & \text{if rand}\left(\right)\leq f\left(p_{ij}^{G}\right)\\ 0, & \text{otherwise,} \end{array}\right. \end{array}$$

where *F* is the scaling factor and *b* denotes the bandwidth factor which is a positive real constant; *p*_*r*1,*j*_^*G*^, *p*_*r*2,*j*_^*G*^, and *p*_*r*3,*j*_^*G*^ are the j-th bits of three randomly chosen individuals of *G* generation. rand() is random number; *u*_*ij*_^′*G*^ is the mutation of the current target individual according to the probability estimation vector *f*(*p*_*ij*_^*G*^).

Crossover operator: The crossover operator is used to produce the trailing individual by mixing the target individual and its mutant individual in MBDE. The trail vector *v*_*ij*_^′*G*+1^ can be obtained as

(10) $$\begin{array}{c} v_{ij}^{\prime G}=\left\{\begin{array}{cc} u_{ij}^{\prime G}, & \text{if }\left(\text{rand}\left(\right)\leq CR\right)\text{ or }\left(j=\text{rand }i\right),\\ p_{ij}^{G}, & \text{otherwise,} \end{array}\right. \end{array}$$

where *v*_*ij*_′ is the element of the trailing individual *v*_*i*_′ and *CR* is the crossover probability ranged (0,1). The rand() is a stochastic number uniformly distributed within (0,1); rand *i* is a random integer with 1,2,…, *N* where *N* is the length of the individual.

The article "Differential Human Learning Optimization Algorithm" was published in 2022. Journal: Comput Intell Neurosci.

Selection: The selection operator is defined as the following equation:

(11) $$\begin{array}{c} x_{i}^{G+1}=\left\{\begin{array}{cc} v_{i}^{G+1}, & \text{if }f\left(v_{i}^{G+1}\right)<f\left(x_{i}^{G}\right),\\ x_{i}^{G}, & \text{otherwise.} \end{array}\right. \end{array}$$

As shown in (11), the MBDE reserved the selection operator of the standard DE. The trail individual *v*_*i*_ replaces the target individual *x*_*i*_ if its fitness value is better. Otherwise, the target individual is reserved for the next generation.

## 3. Differential Human Learning Optimization Algorithm

The three operators of HLO represent human learning randomly, learning from their own experience, and collective experience. However, people could learn from other excellent individuals in actual life. The operator of Differential Evolution (DE) is updated based on the optimal information of other individuals in the population. Inspired by this thought, this paper proposes the differential human learning optimization algorithm (DEHLO), in which the learning strategy of the MBDE is introduced into the HLO to develop a novel probability estimation operator for generating the offspring individuals. And this paper modified the HLO from two levels, i.e., individual and population, and named DEHLO1 and DEHLO2, respectively.

### 3.1. DEHLO1

During the real learning process, different teams always adopt different strategies to search for the optimal solution for the same complex problem. To emulate the phenomena of dividing into groups, the operators of HLO and MBDE are utilized to generate the new solution in DEHLO1, so that the DEHLO1 algorithm could obtain the performance of HLO and MBDE. In DEHLO1, half of the population is updated by using the operator of HLO as (7) to generate a new solution, and the rest of the population is updated by using the mutation operator of MBDE as equations (8)–(10) to acquire the new individual. The DEHLO1 algorithm could possess both the advantages and shortcomings of the HLO and MBDE, and a dynamic competition strategy is used in DEHLO1 to avoid the disadvantages of the HLO and MBDE. At the beginning of a search, the population is divided into two equal parts which adopt the strategy of HLO and MBDE, respectively. With the progress of the search, the optimal fitness of the HLO and that of MBDE are compared under the specified iterations, and the individual proportion of better fitness value corresponding algorithm will be increased while the individual proportion of the other algorithm will be decreased correspondingly. Therefore, the DEHLO1 algorithm can adaptively compete and use the optimal learning strategy to search for the optimal solution, which effectively enhances the optimization ability of the algorithm. The procedure of DEHLO1 can be illustrated in Figure 1.

The article "Differential Human Learning Optimization Algorithm" was published in 2022. Journal: Comput Intell Neurosci.

### 3.2. DEHLO2

In real society, the same problem could be solved by using different approaches. But there might be a mainstream method in a certain period, and the mainstream method might be switched to another method due to the needs of the problem. Exactly as the way of human learning: “practice, knowledge, again practice, and again knowledge” [52], this form repeats itself in endless cycles, and with each cycle, the content of practice and knowledge rises to a higher level. This learning process is a vivid metaphor for the spiral. In DEHLO2, the HLO and the MBDE on the whole population are mixed and executed alternately by mimicking these learning behaviors. Firstly, the entire population adopts the HLO algorithm to search for the optimal solution. If it cannot be updated after a specified iteration, the learning process of HLO will be considered to encounter the bottleneck; then the strategy of MBDE will be executed, which might make the algorithm escape from the bottleneck and vice versa: if the MBDE algorithm cannot find the optimal solution after certain iterations, the HLO algorithm will be executed to update the individual of the population. The flowchart of DEHLO2 is shown in Figure 2.

The procedure of DEHLO2 can be described as follows:

Step 1: Set control parameters, including the population size (popSize), the maximum generation (*G*_max_), the iterations of the search strategy, and the control parameters of HLO and MBDE; Step 2: Initialize the population randomly, calculate the fitness of each individual, and initialize the IKD and SKD; Step 3: Update the individual of the population as equations (8)–(11) of the MBDE algorithm; when the global optimal of MBDE cannot update after the set iterations, use the HLO algorithm to update the individual of the population as equation (7), and so forth, to generate the new population; Step 4: Calculate the fitness of the new individual and update the IKD and SKD; Step 5: If the terminal conditions are met, terminate the iteration; otherwise go to step 3; Step 6: Output the optimal solution.

The article "Differential Human Learning Optimization Algorithm" was published in 2022. Journal: Comput Intell Neurosci.

### 3.3. Algorithm Complexity

DEHLO1 and DEHLO2 both have two phases, i.e., the population initialization and the iterative search. The running times of generating the initial population *X*, individual knowledge database (IKD), and social knowledge database (SKD) are *N* × *M*, *N* × *M*, and (*M*+log  *N*), respectively, where *M* and N represent the dimension of solutions and the size of the population, respectively. So, the overall running time of the population initialization is ((2*N*+1) × *M*+log  *N*). During the iterative search of DEHLOs, generating new individuals costs time *N* × *M*, performing crossover operation costs time *N* × *M*, and updating the IKD and SKD costs times *N* × (*M*+log  *K*) and (log  *N*+log  *S*+*M*), respectively, where K is the predefined number of solutions saved in the IKD and S denotes the size of the SKD. Therefore, the running time of each iterative step is ((3*N*+1) × *M*+log(*N* × *S* × *K*^*N*^)). Assume that the maximum generation of DEHLOs algorithms is *G*, so the iterative search phase takes time *G* × ((3*N*+1) × *M*+log(*N* × *S* × *K*^*N*^)). In general, the maximum generation *G* is much greater than N, K, and S, and therefore the time complexity of DEHLOs is *O*((3*N*+1) × *G* × *M*).

## 4. Experimental Results and Discussions

To verify the performance of the two algorithms, i.e., DEHLO1 and DEHLO2, the proposed DEHLOs as well as other six binary-coding optimization algorithms, i.e., Improved Adaptive Human Learning Optimization (IAHLO) [37], Simple Human Learning Optimization (SHLO) [34], Modified Binary Differential Evolution (MBDE) [47], Novel Binary Differential Evolution (NBDE) [53], Improved Binary Particle Swarm Optimization (IBPSO) [54], and Novel Binary Gaining Sharing Knowledge-based optimization (NBGSK) [17], were applied to solve multidimensional knapsack problems [55]. The parameters pr, pi, CR, F, and *b* adopt the default values of HLO and MBDE, and a set of fair parameters, i.e., Cn and K of DEHLO1 and NM and NH of DEHLO2, is chosen for DEHLO1 and DEHLO2 by trial and error in this paper, that is, Cn = 100, *K* = 5%, NM = 100, and NH = 50. For a fair comparison, the recommended parameters of all compared algorithms were used to tackle the problem, which is listed in Table 1. Since DEHLOs are designed for solving “single-objective” problems, the sizes of IKDs and SKD are both set to 1 [35] to enhance search efficiency and reduce the cost of computation. Besides, the IKD of DEHLOs was reinitialized to further enhance the diversity if it is not updated in the successive 100 generations. The computations were carried out using a PC with Intel Core i5-6402P @ 2.8 GHz CPU and 8 GB RAM while running Java 1.70 on Windows 8.1, 64-bit operating system.

The article "Differential Human Learning Optimization Algorithm" was published in 2022. Journal: Comput Intell Neurosci.

### 4.1. A Set of Multidimensional Knapsack Problems

Knapsack problems have been studied intensively in the last few decades, and multidimensional knapsack problems (MKPs) [55] are multiconstrained problems instead of only one constraint. It can be formulated as

(12) $$\begin{array}{c} \text{Max}f\left(x_{1},x_{2},\ldots ,x_{n}\right)=\sum_{j=1}^{n}p_{j}x_{j},\\ \text{s.t.}\left\{\begin{array}{c} \sum_{j=1}^{n}w_{j}x_{j}\leq C\\ x_{j}\in \left\{0,1\right\},\;j\in \left\{1,2,\ldots ,n\right\}, \end{array}\right. \end{array}$$

where the binary decision variables *x*_*j*_ are used to indicate whether the item *j* is included in the knapsack or not. Without loss of generality, knapsack problems assume that all profits and weights are positive and all the weights are smaller than the capacity *C*. Since the maximal volume of the knapsack is limited in knapsack problems and the total volume of the items packed in the knapsack may exceed the constraint, the violation is unacceptable and must be checked. Thus, the penalty function method as (13) is adopted to deal with the infeasible solutions,

(13) $$\begin{array}{c} \text{Max}F\left(x\right)=\sum_{j=1}^{n}p_{j}x_{j}-\beta \cdot \max\left(0,\sum_{j=1}^{n}w_{j}x_{j}-C\right),\\ \text{s.t.}x_{j}\in \left\{0,1\right\},\;j=1,2,\ldots ,n, \end{array}$$

where the penalty coefficient *β* is a big constant which can lead the algorithm to escape from the infeasible area.

For a comprehensive comparison, a total of 30 multidimensional knapsack problems (MKPs), i.e., the instances 5.250.00-29, are adopted to test the performance of DEHLOs as well as the other metaheuristics. The population size and the maximum generation of all the algorithms are set to 100 and 5000. Four indicators, i.e., the best fitness value (Best), the mean best fitness value (Mean), the worst fitness value (Worst), and the standard deviation (Std), are used to evaluate the performance of DEHLOs. Each algorithm ran 100 times on all the problems independently. The numerical results are given in Table 2.

To better compare the performance of DEHLOs with other algorithms, the results of student's *t*-test (*t*-test) and Wilcoxon signed-rank test (W-test) are also listed in Table 2 where “1” indicates that DEHLO2 is significantly better than the compared algorithms at the 95% confidence, “−1” represents that DEHLO2 is significantly worse than the compared algorithms, and “0” denotes that the performance of DEHLO2 is equivalent to other algorithms. Note that the *t*-test, a parameter test, needs to satisfy the normality and homogeneity of variance, while the W-test, a nonparametric test, does not need. Therefore, the *t*-test is more reliable when the Gaussian distribution assumption is met while the W-test would be more powerful when this assumption is violated [35]. For convenience, the results of the *t*-test and W-test are summarized in Table 3.

The article "Differential Human Learning Optimization Algorithm" was published in 2022. Journal: Comput Intell Neurosci.

Table 2 shows that the proposed DEHLO2 obtains the best numerical results on 26 out of 30 instances. Besides, the summary results of the *t*-test show that DEHLO2 is obviously better than DEHLO1, IAHLO, HLO, MBDE, NBDE, IBPSO, and NBGSK on 21, 30, 30, 24, 30, 30, and 30 out of 30 instances. And W-test results also show that DEHLO2 is significantly superior to DEHLO1, IAHLO, HLO, MBDE, NBDE, IBPSO, and NBGSK on 21, 30, 30, 23, 30, 30, and 30 out of 30 instances. Based on Tables 2 and 3, it is fair to say that DEHLO2 outperforms other algorithms on the multidimensional knapsack problems.

### 4.2. Another Set of Multidimensional Knapsack Problems

To further verify the performance of the proposed algorithm, another set of multidimensional knapsack problems [53] is adopted as the test benchmark, which is listed in Table 4. The results of all algorithms on the MKPs are given in Table 5 where the best solutions have been highlighted in bold. And the summary results of the *t*-test and W-test are summarized in Table 6. To analyze the superiority of the proposed DEHLOs, the convergence curves of all algorithms on the MKPs are drawn in Figure 3.

It can be seen from Tables 5 and 6 and Figure 3 that DEHLO2 provides the best results and obtained the minimum error among the other algorithms. Specifically, DEHLO2 attains the best numerical results on 13 out of 14 instances and is only inferior to DEHLO1 on the instance 5.500.01. The summarized *t*-test and W-test results indicate that the proposed DEHLO2 significantly surpasses IAHLO, HLO, MBDE, NBDE, IBPSO, and NBGSK on all the instances while it is better than, competitive to, and worse than DEHLO1 on 10, 4, and 0 instances on the *t*-test and 11, 3, and 0 instances on the *W*-test, respectively. Furthermore, Figure 3 shows that the proposed DEHLOs algorithm has a faster convergence rate and higher solution accuracy than the compared algorithms. Therefore, with the introduction of the strategy of MBDE, the optimization performance of the DEHLOs algorithm is significantly enhanced.

## 5. Conclusions and Future Work

Human learning optimization is a simplified model of human learning; it develops three learning operators, i.e. the random learning operator, the individual learning operator, and the social learning operator, to search for the optimal solution. However, the standard HLO just learns from the global optimal solution; this is inconsistent with reality. In real life, people can learn from the optimal solution of other individuals. And the operators of Differential Evolution (DE) are updated based on the optimal solution of other individuals. Inspired by this fact, this paper introduces the optimization strategy of MBDE into HLO and presents two novel differential human learning optimization algorithms based on individual and population. To comprehensively and fairly evaluate the performance of proposed algorithms, the multidimensional knapsack problems were adopted as the benchmark problems to test DEHLOs, as well as the standard HLO, MBDE, and other metaheuristics. The experimental results demonstrate that the proposed DEHLOs can utilize the learning ability of the two algorithms to search for the optimal solution more efficiently and have a robust search ability for different problems.

The article "Differential Human Learning Optimization Algorithm" was published in 2022. Journal: Comput Intell Neurosci.

It is well known that humans can adaptively choose and adjust these approaches to solve problems efficiently and effectively. However, the impact of adaptive learning strategy on algorithm parameters is not considered in this paper. Therefore, one of our future works is to develop adaptive switching learning strategies to better release the power of different learning strategies for different problems, which will be very challenging for future work.

## Figures and Tables

**Figure 1:** The flowchart of DEHLO1.

**Figure 2:** The flowchart of DEHLO2.

**Figure 3:** The convergence curves of the MKP (maximum generation = 5000).

**Algorithm 1:** Pseudocode of HLO.

**Table 1:** The recommended parameter values of all the algorithm.

Algorithm	Parameters settings
DEHLO1	*pr* = 5/*M*, *pi* = 0.85 + 2/*M*, CR = 0.2, *F* = 0.8, *b* = 20, Cn = 100, *K* = 5%
DEHLO2	*pr* = 5/*M*, *pi* = 0.85 + 2/*M*, CR = 0.2, *F* = 0.8, *b* = 20, NM = 100, NH = 50
IAHLO [37]	*pr*_min1_ = 0.02, *pr*_min2_ = 0.05, *pr*_max_ = 0.15, *pi* = 0.85 + 2/*M*, Sp = 0.2 × *G*_max_
SHLO [34]	*pr* = 5/*M*, *pi* = 0.85 + 2/*M*
MBDE [47]	CR = 0.2, *F* = 0.8, *b* = 20
NBDE [53]	*F* = 1.0, CR = 0.5, filp = 0.2, *U*_min_ = 0.1 × *M*, *U*_max_ = 0.9 × *M*
IBPSO [54]	*ω*min = 0.0, *ω*max = 2.0, *c*1 = 1.75, *c*2 = 2.00, *V*_min_ = −6, *V*_max_ = 6
NBGSK [17]	NP_min_ = 12, Np_max_ = 200, *k*_*f*_ = 1.0, *k*_*r*_ = 0.9, *p* = 0.1, *δ* = 100, *λ* = −100

*Note. M* is the dimension of solutions.

**Table 2:** The results of all algorithms on the multidimensional knapsack problems.

Problem	Algorithm	Best	Mean	Worst	Std	*t*-test	*W*-test
5.250.0	DEHLO2	59208	59071.35	58968	45.81	—	—
	DEHLO1	59196	59054.47	58941	46.52	1	1
	IAHLO	58541	58145.82	57831	130.21	1	1
	SHLO	59170	58990.19	58845	65.47	1	1
	MBDE	58900	58765.98	58643	47.17	1	1
	NBDE	58745	58269.03	57715	229.58	1	1
	IBPSO	58935	58521.45	57942	188.27	1	1
	NBGSK	57486	56579.44	55336	411.20	1	1

5.250.1	DEHLO2	61446	61381.94	61268	50.44	—	—
	DEHLO1	61377	61308.04	61209	46.25	1	1
	IAHLO	60550	60117.68	59695	158.28	1	1
	SHLO	61435	61274.52	61138	62.09	1	1
	MBDE	61139	61096.41	60969	40.32	1	1
	NBDE	61078	60269.88	59566	380.60	1	1
	IBPSO	61213	60795.96	60073	214.59	1	1
	NBGSK	59324	58075.21	56888	516.38	1	1

5.250.2	DEHLO2	62057	61959.72	61876	45.92	—	—
	DEHLO1	62028	61946.21	61855	43.06	1	1
	IAHLO	61013	60599.87	60309	154.33	1	1
	SHLO	62008	61865.90	61682	54.89	1	1
	MBDE	62057	61937.51	61850	41.77	1	1
	NBDE	61417	60780.85	60265	225.67	1	1
	IBPSO	61640	61166.56	60485	240.18	1	1
	NBGSK	60205	59110.06	58296	395.35	1	1

5.250.3	DEHLO2	59343	59235.19	59143	39.21	—	—
	DEHLO1	59315	59233.84	59123	41.67	0	0
	IAHLO	58615	58294.18	58042	117.85	1	1
	SHLO	59304	59162.28	58988	61.14	1	1
	MBDE	59334	59238.46	59158	40.94	0	0
	NBDE	58760	58388.26	57986	184.56	1	1
	IBPSO	59168	58752.84	58406	163.98	1	1
	NBGSK	57855	57014.16	56243	340.69	1	1

5.250.4	DEHLO2	58913	58799.33	58665	44.29	—	—
	DEHLO1	58935	58791.13	58696	47.27	0	0
	IAHLO	57865	57540.15	57145	143.82	1	1
	SHLO	58878	58703.24	58564	60.21	1	1
	MBDE	58877	58758.46	58631	44.55	1	1
	NBDE	58176	57666.00	57090	239.22	1	1
	IBPSO	58608	58171.05	57670	190.88	1	1
	NBGSK	56972	55896.45	55107	417.30	1	1

5.250.5	DEHLO2	60005	59884.27	59786	43.45	—	—
	DEHLO1	59980	59865.34	59752	52.38	1	1
	IAHLO	58760	58457.12	57975	149.44	1	1
	SHLO	59969	59784.46	59645	65.58	1	1
	MBDE	59945	59842.43	59696	47.81	1	1
	NBDE	59220	58724.95	58246	209.78	1	1
	IBPSO	59714	59151.86	58576	258.90	1	1
	NBGSK	58032	56999.98	56025	441.22		

5.250.6	DEHLO2	60363	60300.41	60222	29.38	—	—
	DEHLO1	60358	60281.02	60199	32.38	1	1
	IAHLO	59378	58953.02	58536	163.95	1	1
	SHLO	60353	60221.83	59964	58.84	1	1
	MBDE	60341	60295.39	60216	31.27	0	0
	NBDE	59968	59306.75	58585	334.58	1	1
	IBPSO	60128	59697.42	58954	210.21	1	1
	NBGSK	58256	57192.39	55838	529.42	1	1

5.250.7	DEHLO2	61443	61364.97	61258	38.19	—	—
	DEHLO1	61443	61354.31	61227	45.12	0	0
	IAHLO	60401	60031.70	59625	147.33	1	1
	SHLO	61443	61276.94	61141	61.80	1	1
	MBDE	61443	61329.16	61185	45.60	1	1
	NBDE	60741	60127.33	59586	285.43	1	1
	IBPSO	61195	60793.69	60209	183.45	1	1
	NBGSK	59397	58110.16	57055	496.41	1	1

5.250.8	DEHLO2	61885	61783.26	61698	37.56	—	—
	DEHLO1	61873	61776.09	61688	38.60	0	0
	IAHLO	60832	60330.40	59847	192.49	1	1
	SHLO	61849	61711.02	61579	53.10	1	1
	MBDE	61831	61750.80	61627	36.37	1	1
	NBDE	61332	60640.49	59841	293.99	1	1
	IBPSO	61626	61116.24	60530	208.09	1	1
	NBGSK	59896	58378.40	57110	608.34	1	1

5.250.9	DEHLO2	58906	58825.17	58768	26.75	—	—
	DEHLO1	58915	58818.13	58755	31.43	0	0
	IAHLO	58085	57822.15	57505	127.82	1	1
	SHLO	58865	58759.37	58618	51.08	1	1
	MBDE	58918	58831.57	58695	43.94	0	0
	NBDE	58651	58235.22	57531	240.98	1	1
	IBPSO	58803	58407.19	57940	165.90	1	1
	NBGSK	57454	56359.20	55279	444.44	1	1

5.250.10	DEHLO2	109031	108945.41	108878	35.61	—	—
	DEHLO1	109051	108935.47	108850	37.12	0	0
	IAHLO	108164	107737.36	107401	157.60	1	1
	SHLO	109013	108879.42	108723	49.85	1	1
	MBDE	109047	108930.03	108875	29.74	1	1
	NBDE	108652	108235.63	107873	188.02	1	1
	IBPSO	108820	108358.03	107786	183.12	1	1
	NBGSK	107078	105016.71	102248	830.71	1	1

5.250.11	DEHLO2	109788	109724.02	109671	30.13	—	—
	DEHLO1	109821	109715.09	109620	34.97	0	0
	IAHLO	108832	108389.65	108106	157.90	1	1
	SHLO	109778	109643.79	109526	55.61	1	1
	MBDE	109821	109731.71	109666	33.94	0	0
	NBDE	109407	109035.96	108574	182.36	1	1
	IBPSO	109498	109134.90	108575	203.18	1	1
	NBGSK	107415	105664.99	102848	960.86	1	1

5.250.12	DEHLO2	108480	108421.36	108341	31.26	—	—
	DEHLO1	108481	108391.59	108271	44.11	1	1
	IAHLO	107602	107248.20	106838	147.38	1	1
	SHLO	108472	108308.74	108154	63.91	1	1
	MBDE	108504	108402.61	108317	36.50	1	1
	NBDE	108108	107752.60	107255	177.67	1	1
	IBPSO	108202	107802.48	107355	188.54	1	1
	NBGSK	106129	104260.07	101348	956.81	1	1

5.250.13	DEHLO2	109352	109291.79	109229	28.48	—	—
	DEHLO1	109356	109279.64	109210	31.72	1	1
	IAHLO	108392	108113.52	107871	117.43	1	1
	SHLO	109325	109220.67	109081	45.88	1	1
	MBDE	109351	109276.32	109208	31.63	1	1
	NBDE	109124	108621.42	108222	192.78	1	1
	IBPSO	109113	108650.60	107755	230.00	1	1
	NBGSK	107356	105919.36	104001	825.83	1	1

5.250.14	DEHLO2	110654	110559.06	110476	37.70	—	—
	DEHLO1	110639	110537.86	110459	35.69	1	1
	IAHLO	109510	109124.47	108774	150.24	1	1
	SHLO	110602	110469.79	110342	56.66	1	1
	MBDE	110632	110553.12	110462	33.98	0	0
	NBDE	110256	109752.20	109320	231.02	1	1
	IBPSO	110359	109948.59	109246	222.17	1	1
	NBGSK	108155	106374.74	104159	818.68	1	1

5.250.15	DEHLO2	110202	110108.40	110006	36.40	—	—
	DEHLO1	110191	110092.18	109992	42.80	1	1
	IAHLO	109213	108875.59	108564	125.81	1	1
	SHLO	110136	110005.03	109797	58.11	1	1
	MBDE	110175	110078.90	110001	40.38	1	1
	NBDE	109892	109405.00	108941	221.35	1	1
	IBPSO	109885	109526.95	108827	227.84	1	1
	NBGSK	107897	106311.66	103800	828.51	1	1

5.250.16	DEHLO2	108990	108921.89	108852	29.26	—	—
	DEHLO1	109002	108905.32	108811	33.75	1	1
	IAHLO	107916	107558.11	107196	146.05	1	1
	SHLO	108987	108837.38	108712	52.22	1	1
	MBDE	109002	108914.46	108837	25.72	1	0
	NBDE	108638	108251.11	107792	185.92	1	1
	IBPSO	108741	108383.70	107829	186.15	1	1
	NBGSK	106606	105029.12	103040	813.45	1	1

5.250.17	DEHLO2	108978	108880.64	108798	38.02	—	—
	DEHLO1	108979	108875.64	108794	40.73	0	0
	IAHLO	107931	107553.41	107164	154.42	1	1
	SHLO	108942	108807.05	108662	58.16	1	1
	MBDE	108931	108861.85	108756	33.72	1	1
	NBDE	108555	108011.37	107658	197.88	1	1
	IBPSO	108695	108306.38	107821	190.34	1	1
	NBGSK	106414	104892.29	102497	910.07	1	1

5.250.18	DEHLO2	109944	109831.24	109759	33.43	—	—
	DEHLO1	109908	109821.03	109746	37.57	0	0
	IAHLO	109171	108759.55	108514	122.98	1	1
	SHLO	109858	109722.03	109575	62.95	1	1
	MBDE	109956	109814.82	109654	57.86	1	1
	NBDE	109703	109325.19	108829	164.61	1	1
	IBPSO	109647	109241.38	108573	212.85	1	1
	NBGSK	108304	106184.02	103343	1013.96	1	1

5.250.19	DEHLO2	107023	106945.49	106871	27.69	—	—
	DEHLO1	106999	106927.56	106833	27.89	1	1
	IAHLO	106167	105667.04	105270	154.47	1	1
	SHLO	107009	106872.17	106786	49.62	1	1
	MBDE	107023	106952.87	106844	27.00	0	0
	NBDE	106694	106226.87	105724	248.58	1	1
	IBPSO	106679	106364.73	105897	181.83	1	1
	NBGSK	104423	102663.29	99947	962.96	1	1

5.250.20	DEHLO2	149623	149543.31	149484	29.41	—	—
	DEHLO1	149634	149533.39	149468	34.64	1	1
	IAHLO	148681	148320.02	147978	140.74	1	1
	SHLO	149573	149470.07	149382	41.14	1	1
	MBDE	149539	149342.64	149032	110.93	1	1
	NBDE	148884	148622.34	148307	123.10	1	1
	IBPSO	149306	148955.74	148331	181.61	1	1
	NBGSK	147760	146521.63	143993	672.83	1	1

5.250.21	DEHLO2	155940	155897.43	155838	23.65	—	—
	DEHLO1	155944	155875.40	155806	30.46	1	1
	IAHLO	155065	154738.49	154326	144.47	1	1
	SHLO	155890	155820.99	155677	41.30	1	1
	MBDE	155898	155721.54	155461	99.55	1	1
	NBDE	155431	155258.09	154912	91.96	1	1
	IBPSO	155691	155382.19	154855	175.20	1	1
	NBGSK	154255	152302.20	150353	840.25	1	1

5.250.22	DEHLO2	149301	149239.94	149187	27.44	—	—
	DEHLO1	149301	149218.06	149147	32.76	1	1
	IAHLO	148471	148143.82	147699	146.26	1	1
	SHLO	149301	149172.26	149075	45.63	1	1
	MBDE	149229	149013.95	148749	114.15	1	1
	NBDE	148639	148381.64	147994	137.00	1	1
	IBPSO	149091	148772.64	148339	160.97	1	1
	NBGSK	147441	146336.57	144699	605.23	1	1

5.250.23	DEHLO2	152130	152084.27	152009	20.64	—	—
	DEHLO1	152124	152070.18	151999	24.23	1	1
	IAHLO	151098	150707.83	150292	169.01	1	1
	SHLO	152114	152007.41	151871	49.62	1	1
	MBDE	152073	151899.50	151719	90.65	1	1
	NBDE	151686	151389.37	150953	159.61	1	1
	IBPSO	151898	151463.97	151054	178.66	1	1
	NBGSK	150151	148785.67	146882	693.66	1	1

5.250.24	DEHLO2	150353	150297.60	150229	20.04	—	—
	DEHLO1	150351	150277.77	150199	30.33	1	1
	IAHLO	149405	148986.69	148598	153.20	1	1
	SHLO	150310	150235.86	150136	40.98	1	1
	MBDE	150353	150096.92	149785	137.68	1	1
	NBDE	149678	149484.92	149221	103.73	1	1
	IBPSO	150095	149672.29	148886	212.06	1	1
	NBGSK	148524	146966.44	145005	709.20	1	1

5.250.25	DEHLO2	150045	149978.52	149870	31.92	—	—
	DEHLO1	150045	149954.51	149868	38.76	1	1
	IAHLO	149308	148912.90	148632	131.50	1	1
	SHLO	149983	149871.36	149720	53.00	1	1
	MBDE	149918	149742.86	149387	99.89	1	1
	NBDE	149352	149183.69	148878	83.20	1	1
	IBPSO	149895	149532.97	148973	165.35	1	1
	NBGSK	148482	147229.26	144434	827.86	1	1

5.250.26	DEHLO2	148574	148507.49	148446	24.57	—	—
	DEHLO1	148553	148499.85	148425	28.71	1	1
	IAHLO	147764	147416.29	147078	146.96	1	1
	SHLO	148542	148445.73	148306	46.31	1	1
	MBDE	148512	148362.46	148147	91.14	1	1
	NBDE	148199	147972.07	147504	106.02	1	1
	IBPSO	148405	148015.40	147518	206.74	1	1
	NBGSK	146709	145373.45	143358	782.85	1	1

5.250.27	DEHLO2	149767	149746.97	149714	14.04	—	—
	DEHLO1	149782	149736.77	149684	20.57	1	1
	IAHLO	148940	148436.47	147929	186.75	1	1
	SHLO	149767	149694.35	149579	36.13	1	1
	MBDE	149767	149523.50	149257	103.60	1	1
	NBDE	148887	148601.80	148006	185.60	1	1
	IBPSO	149628	149230.72	148773	172.73	1	1
	NBGSK	147575	146086.06	144103	771.83	1	1

5.250.28	DEHLO2	155075	155012.04	154961	25.70	—	—
	DEHLO1	155075	154993.48	154914	31.91	1	1
	IAHLO	154135	153707.79	153291	165.97	1	1
	SHLO	155029	154927.58	154814	38.04	1	1
	MBDE	155032	154900.12	154715	69.24	1	1
	NBDE	154664	154414.09	153963	144.58	1	1
	IBPSO	154806	154514.11	153986	160.66	1	1
	NBGSK	153292	151840.26	149513	704.28	1	1

5.250.29	DEHLO2	154668	154640.60	154590	17.70	—	—
	DEHLO1	154668	154623.56	154542	21.97	1	1
	IAHLO	153751	153406.13	153011	140.95	1	1
	SHLO	154668	154562.83	154434	52.21	1	1
	MBDE	154653	154460.96	154239	76.42	1	1
	NBDE	154298	154056.73	153720	108.12	1	1
	IBPSO	154641	154136.17	153595	209.88	1	1
	NBGSK	152952	151403.32	148808	859.73	1	1

The article "Differential Human Learning Optimization Algorithm" was published in 2022. Journal: Comput Intell Neurosci.

**Table 3:** The summary results of the *t*-test and W-test on multidimensional knapsack problems.

Metric	DEHLO2	DEHLO1	IAHLO	SHLO	MBDE	NBDE	IBPSO	NBGSK
*t*-test	1	21	30	30	24	30	30	30
	0	9	0	0	6	0	0	0
	−1	0	0	0	0	0	0	0

*W*-test	1	21	30	30	23	30	30	30
	0	9	0	0	7	0	0	0
	−1	0	0	0	0	0	0	0

**Table 4:** The multidimensional knapsack problem benchmarks.

Benchmark NO.	Benchmark name	Best known	*n*	*M*
1	mknapcb1–5.100–00	244381	100	5
2	mknapcb1–5.100–01	24274	100	5
3	mknapcb2–5.250–00	59312	250	5
4	mknapcb2–5.250–01	61472	250	5
5	mknapcb3–5.500–00	120130	500	5
6	mknapcb3–5.500–01	117837	500	5
7	mknapcb4–10.100–00	23064	100	10
8	mknapcb4–10.100–01	22801	100	10
9	mknapcb5–10.250–00	59187	250	10
10	mknapcb5–10.250–01	58662	250	10
11	mknapcb6–10.500–00	117726	500	10
12	mknapcb6–10.500–01	119139	500	10
13	mknapcb8–30.250–29	150038	250	30
14	mknapcb9–30.500–29	301021	500	30

**Table 5:** The results of all algorithms on the multidimensional knapsack problems.

Problem	Algorithm	Best	Mean	Worst	Std	*t*-test	*W*-test
NO.1	DEHLO2	24381	24373.92	24337	8.95	—	—
	DEHLO1	24381	24364.37	24315	18.76	1	1
	IAHLO	24381	24297.24	24187	41.30	1	1
	SHLO	24357	24347.09	24292	14.41	1	1
	MBDE	24332	24327.72	24288	6.59	1	1
	NBDE	24381	24285.06	24185	42.22	1	1
	IBPSO	24381	24177.04	23862	106.18	1	1
	NBGSK	24047	23721.87	23395	140.08	1	1

NO.2	DEHLO2	24274	24274.00	24274	0.00	—	—
	DEHLO1	24274	24262.90	24149	35.50	1	1
	IAHLO	24274	24136.40	23911	89.93	1	1
	SHLO	24250	24243.75	24125	27.38	1	1
	MBDE	24225	24222.67	24101	16.43	1	1
	NBDE	24274	24194.46	23878	95.50	1	1
	IBPSO	24274	23964.76	23575	143.60	1	1
	NBGSK	23893	23388.82	22930	174.22	1	1

NO.3	DEHLO2	59208	59071.35	58968	45.81	—	—
	DEHLO1	59196	59054.47	58941	46.52	1	1
	IAHLO	58541	58145.82	57831	130.21	1	1
	SHLO	59170	58990.19	58845	65.47	1	1
	MBDE	58900	58765.98	58643	47.17	1	1
	NBDE	58745	58269.03	57715	229.58	1	1
	IBPSO	58935	58521.45	57942	188.27	1	1
	NBGSK	57486	56579.44	55336	411.20	1	1

NO.4	DEHLO2	61446	61381.94	61268	50.44	—	—
	DEHLO1	61377	61308.04	61209	46.25	1	1
	IAHLO	60550	60117.68	59695	158.28	1	1
	SHLO	61435	61274.52	61138	62.09	1	1
	MBDE	61139	61096.41	60969	40.32	1	1
	NBDE	61078	60269.88	59566	380.60	1	1
	IBPSO	61213	60795.96	60073	214.59	1	1
	NBGSK	59324	58075.21	56888	516.38	1	1

NO.5	DEHLO2	119661	119457.17	119243	75.81	—	—
	DEHLO1	119588	119409.80	119223	80.53	0	0
	IAHLO	116330	115483.56	114961	249.75	1	1
	SHLO	119582	119303.70	119008	110.02	1	1
	MBDE	119372	119153.95	118985	93.96	1	1
	NBDE	116080	115220.19	114501	406.61	1	1
	IBPSO	118959	118292.17	117429	361.22	1	1
	NBGSK	115208	112449.12	111021	919.05	1	1

NO.6	DEHLO2	117579	117494.62	117356	44.63	—	—
	DEHLO1	117662	117498.59	117359	54.85	1	1
	IAHLO	114647	113959.66	113396	248.20	1	1
	SHLO	117543	117345.74	117099	89.98	1	1
	MBDE	117501	117326.38	117141	80.53	1	1
	NBDE	115477	113941.85	112855	586.89	1	1
	IBPSO	116956	116314.68	115314	330.61	1	1
	NBGSK	113416	111349.51	109234	887.34	1	1

NO.7	DEHLO2	23064	23054.91	23026	3.19	—	—
	DEHLO1	23057	23052.57	22959	11.49	0	1
	IAHLO	23055	23040.13	22901	36.68	1	1
	SHLO	23041	23032.01	23027	1.17	1	1
	MBDE	23018	23009.34	23009	1.36	1	1
	NBDE	23064	23029.70	22845	51.32	1	1
	IBPSO	23055	22863.90	22574	117.69	1	1
	NBGSK	22876	22593.57	22282	113.85	1	1

NO.8	DEHLO2	22801	22714.70	22541	60.08	—	—
	DEHLO1	22801	22713.56	22547	60.03	0	0
	IAHLO	22739	22517.76	22344	78.27	1	1
	SHLO	22801	22690.79	22502	79.50	1	1
	MBDE	22755	22666.18	22539	53.80	1	1
	NBDE	22801	22478.81	22323	77.18	1	1
	IBPSO	22725	22386.50	21994	127.65	1	1
	NBGSK	22422	22067.62	21844	113.60	1	1

NO.9	DEHLO2	59071	58853.87	58679	73.36	—	—
	DEHLO1	59012	58796.65	58614	72.72	1	1
	IAHLO	58309	58031.44	57679	128.93	1	1
	SHLO	59071	58768.92	58551	95.55	1	1
	MBDE	58438	58254.09	58112	54.10	1	1
	NBDE	58410	57849.68	57416	212.98	1	1
	IBPSO	58756	58337.24	57861	182.21	1	1
	NBGSK	57378	56515.92	55741	420.44	1	1

NO.10	DEHLO2	58637	58519.04	58359	62.07	—	—
	DEHLO1	58567	58449.57	58324	53.74	1	1
	IAHLO	57946	57355.51	57014	155.67	1	1
	SHLO	58599	58447.36	58292	70.06	1	1
	MBDE	58596	58457.51	58348	54.78	1	1
	NBDE	57715	57135.82	56790	177.76	1	1
	IBPSO	58277	57812.49	57285	209.48	1	1
	NBGSK	56931	55925.43	55228	289.04	1	1

NO.11	DEHLO2	117149	116895.63	116606	103.48	—	—
	DEHLO1	117001	116672.01	116433	112.36	1	1
	IAHLO	114617	114048.13	113553	230.22	1	1
	SHLO	117194	116847.53	116390	130.52	1	1
	MBDE	116734	116456.38	116209	118.63	1	1
	NBDE	114440	113394.71	112891	300.95	1	1
	IBPSO	116597	115690.33	114316	391.02	1	1
	NBGSK	112953	111386.10	110305	639.62	1	1

NO.12	DEHLO2	118732	118554.12	118281	98.71	—	—
	DEHLO1	118663	118426.25	118216	95.64	1	1
	IAHLO	116171	115720.44	115233	236.82	1	1
	SHLO	118768	118446.03	118100	122.62	1	1
	MBDE	118501	118219.57	118029	103.17	1	1
	NBDE	115669	114706.44	114207	314.98	1	1
	IBPSO	118270	117310.97	116181	383.94	1	1
	NBGSK	115125	112837.49	110855	878.62	1	1

NO.13	DEHLO2	149595	149437.59	149346	42.40	—	—
	DEHLO1	149593	149432.14	149291	49.73	0	0
	IAHLO	148784	148447.93	148047	151.62	1	1
	SHLO	149496	149374.31	149222	63.78	1	1
	MBDE	149510	149352.93	149270	60.66	1	1
	NBDE	149204	148977.35	148506	128.08	1	1
	IBPSO	149249	148737.54	147408	321.85	1	1
	NBGSK	148428	146898.01	144999	821.84	1	1

NO.14	DEHLO2	300152	299931.22	299756	68.23	—	—
	DEHLO1	300093	299889.33	299704	87.69	1	1
	IAHLO	295779	295030.14	294131	367.14	1	1
	SHLO	300070	299778.88	299484	117.69	1	1
	MBDE	300107	299854.78	299698	71.82	1	1
	NBDE	298960	298199.49	295981	600.02	1	1
	IBPSO	299290	298355.63	296002	736.99	1	1
	NBGSK	296573	293231.65	287069	2210.58	1	1

The article "Differential Human Learning Optimization Algorithm" was published in 2022. Journal: Comput Intell Neurosci.

**Table 6:** The summary results of the *t*-test and W-test on multidimensional knapsack problems.

Metric	DEHLO2	DEHLO1	IAHLO	SHLO	MBDE	NBDE	IBPSO	NBGSK
*t*-test	1	10	14	14	14	14	14	14
	0	4	0	0	0	0	0	0
	−1	0	0	0	0	0	0	0

*W*-test	1	11	14	14	14	14	14	14
	0	3	0	0	0	0	0	0
	−1	0	0	0	0	0	0	0

## Data Availability

As the data also form part of an ongoing study, the raw/processed data required to reproduce these findings cannot be shared at this time.
